RETRACTED

# Glucosamine Supplementation in Premating Drinking Water Improves Within-Litter Birth Weight Uniformity of Rats Partly through Modulating Hormone Metabolism and Genes Involved in Implantation

**DOI:** 10.1155/2020/1630890

**Published:** 2020-01-04

**Authors:** Cuiping Feng, Taolin Yuan, Shilan Wang, Ting Liu, Shiyu Tao, Dandan Han, Junjun Wang

**Affiliations:** ^1^Department of Obstetrics and Gynecology, China-Japan Friendship Hospital, Beijing 100029, China; ^2^State Key Laboratory of Animal Nutrition, College of Animal Science and Technology, China Agricultural University, Beijing 100193, China

## Abstract

Within-litter birth weight variation in multiparous animals has become a big issue due to high incidence of low birth weight neonates, which gives rise to high preweaning mortality and morbidity. Foetus with various birth weights is the outcome of diverse embryos competence which is affected by oocyte quality. Glucosamine (GlcN) has been reported to be involved in oocyte maturation; however, its effect on pregnant outcomes remains unknown. The present study was conducted to investigate the effects of premating GlcN supplementation via drinking water on within-litter birth weight variation and its underlying mechanism. Fifty eight Sprague-Dawley female rats were randomly assigned to one of two groups with normal drinking water or drinking water supplemented with 0.5 mM GlcN from six to eight weeks old. Variation of within-litter birth weight in the GlcN group was 5.55%, significantly lower compared with 8.17% in the control group. Birth weight was significantly increased in the GlcN group (2.27 ± 0.06) compared with the control group (2.08 ± 0.04). Both absolute and relative weights of the ovary at the end of GlcN treatment were higher in the GlcN group than in the control group (*P* < 0.05). In the GlcN group, there were more successfully implanted blastocysts (13.38 ± 0.63 and 15.75 ± 0.59 in the control and treatment group, respectively) with more uniform distribution along the two uterine horns compared with the control group. Besides, gene expressions of Alk3 and Bmp2 were increased in the implantation sites, while IGF-1 and Mucin-1 were decreased significantly in rats administrated with GlcN. Maternal progesterone, estradiol, and IGF-1 concentrations on D 19.5 were significantly increased, while insulin and total cholesterol levels were significantly decreased in contrast with control dams. In summary, the administration of 0.5 mM GlcN solution before mating reduced within-litter birth weight variation, accompanied with increased fetal weight. Further investigation indicated that the improved outcome of pregnancy results at least partly from the increased ovary weights of the rats, the homogeneous embryo developmental competence, the enhanced receptivity of the uterine environment, and the adjusted maternal hormone levels.

RETRACTED

## 1. Introduction

Poor postnatal survival and retarded growth performance induced by low birth weight and high within-litter birth weight variation in litter-bearing animals have been recognized for many decades [1, 2]. Birth weight variation can be influenced by many factors including breed, maternal physiology, and nutrition. The external environment of females before and during pregnancy, including nutrient intake, dietary behavior, temperature, and health condition, has a significant influence on oocyte and embryo development [3]. Changes in the amount and composition of food or diet consumed before mating can affect oocyte maturation, blastocyst production, prenatal survival, and the number of surviving offspring [4].

In addition, maternal physiological conditions, especially lipid metabolism and hormones, play important roles in pregnancy results. During oocyte maturation or early embryonic development, diet-induced changes in maternal fatty acids may impact follicles and embryo quality [5]. Fatty acids are precursors of steroids and prostaglandins, and they are important for regular reproductive functions [6].

Exposed mouse cumulus-oocyte complexes to glucosamine (GlcN) during in vitro maturation severely perturbed blastocyst development [7]. Although the roles of GlcN on oocyte maturation and early embryo development have been studied *in vitro*, the effects of GlcN supplementation before mating on embryo implantation and reproductive results are poorly understood. The purpose of this paper was to investigate whether GlcN supplementation before mating improved within-litter birth weight uniformity related to the maternal metabolism and hormone concentration in serum and the expression of genes that target in implantation sites.

## 2. Materials and Methods

### 2.1. Animals, Diet, and Experimental Design

Sprague-Dawley (SD) dams (*n* = 58) were purchased from Sibeifu Inc. (Beijing, China). They were five weeks old and then acclimated for one week. The dams were housed individually at 23°C in a room with a 12 h light/12 h dark cycle and water and feed were provided ad libitum. This study was carried out in accordance with the recommendations of the guidelines for the Institutional Animal Care and Use Committee of China Agricultural University (AW11099102-1, Beijing, China).

The rats were fed a basal diet before mating and the pregnant rats were fed a reproductive diet during pregnancy, both of them mainly including corn, soybean meal, fish meal, flour, wheat bran, calcium ammonium phosphate salt, limestone powder, vitamin, microelements, and amino acids. Diet composition was supplied in the additional file ([Supplementary-material supplementary-material-1]). The supplementation of GlcN (D-(+)-glucosamine, purity ≥99%, Sigma-Aldrich) was achieved via dissolving in drinking water. Rats (*n* = 29 per group) were allocated randomly to either 0.5 mM GlcN solution (the concentration was determined on the basis of a gradient experiment which additionally included 1.0 mM GlcN and the results are presented in [Supplementary-material supplementary-material-1]) or drinking water as control. GlcN treatment lasted for two weeks when the dams were six to eight weeks old. After two-week GlcN administration, each dam was caged overnight with a male SD rat to mate. The presence of sperm in the vaginal smear the next morning was regarded as day 0.5 of pregnancy [8]. Unmated females were recaged with males and GlcN operations were continued until mating was completed, or mating attempts were made for up to 4 nights. Those that had not mated until the 4^th^ night were excluded from the study, as described previously [8]. During GlcN treatment periods, rats were weighed individually at days 1, 5, 10, and 14 before mating. Feed and water consumption were monitored. Average daily gain (ADG), average daily feed intake (ADFI), and average daily drinking water intake (ADWI) were recorded to measure the growth performance of rats.

RETRACTED

### 2.2. Sample Collection

The day before mating was regarded as day−1; 20 female rats (10 for Control and 10 for GlcN) were anesthetized by intraperitoneal injection of 1% sodium pentobarbital at 10 mg/100 g body weight and then sacrificed 5 minutes later. After weighed, ovaries and uteri were frozen in liquid nitrogen as soon as possible and then transformed to −80°C. The relative organ index = organ weight/body weight *∗* 100%. On the 6.5th day of pregnancy, when embryos started to contact the uterine endothelium, eight female rats per group were anaesthetized. Through intravenous injecting (0.1 mL/rat) Chicago Sky Blue dye solution (1% in saline, Sigma-Aldrich), implantation sites were observed according to previous studies [8, 9]. Rats were sacrificed 5 min later as described above, and then implantation sites were recorded and collected for further analysis. Pregnant rats (*n* = 11/group) were sacrificed as described above to investigate reproductive results on day 19.5 of gestation (gestation generally lasts 21–23 days) [8]. Coefficient of pup birth weight variation = standard deviation of litter birth weight/average litter birth weight. Maternal placental efficiency = fetal body weight/placental weight ratio [10]. The plasma of dams was collected in tubes containing anticoagulant from vena cava and then centrifuged at 3,000 rpm for 15 min and stored at −20°C for subsequent analysis.

RETRACTED

### 2.3. RNA Extraction and Quantitative Real-Time PCR Analysis

Total RNA was isolated from implantation sites using Trizol reagent (CWBIO, China) according to the manufacturer's instructions, and RNA quality was determined with a Nano-Drop spectrophotometer (Thermo Scientific, USA). One microgram of RNA was reverse transcribed with RevertAid 1st Strand cDNA Synthesis Kit (Thermo, USA). The sequence of the primers is supplied in [Supplementary-material supplementary-material-1] [11–13], including specific genes ALK3, BMP2, insulin-like growth factor 1 (IGF-1), Mucin-1, iNOS, and *β*-actin. Gene expression of *β*-actin in each sample was quantified as a control. Complementary DNA (cDNA) was then used to amplify these primers by using SYBR Green (Takara, Japan) on an Applied Biosystems 7500 Real-Time PCR System (ABI, USA). The 2^−ΔΔct^ method was used to analyze gene expression levels as previously described [14].

### 2.4. Blood Test

To evaluate maternal metabolic state and body condition, total cholesterol (TC), low-density lipoprotein cholesterol (LDL-C), high-density lipoprotein cholesterol (HDL-C), and triglyceride (TG) in plasma were analyzed in duplicate using an Automatic Biochemistry Analyzer (Hitachi 7020, Japan). Estradiol, progesterone, insulin, and IGF-1 were analyzed by radioimmunoassay kits (Sino-UK Inc, China) [8].

### 2.5. Statistical Analysis

Data are presented as means ± SEM. The data were analyzed with Student's unpaired *t*-test (GraphPad Prism version 7.0). Statistical significance was detected at *P* < 0.05 and a trend at 0.05 < *P* < 0.1. The unit in the statistical analysis individually is 11 dams per group for reproductive results, 8 dams per group for uniformity of implantation, and 10 for the organ index before mating.

## 3. Results

### 3.1. GlcN Supplementation before Mating Decreased Within-Litter Birth Weight Variation of Rats

In the present study, fetal weight refers to body weight in late pregnancy (day 19.5 of pregnancy), since colostrum intake could alter neonatal body weight and the variation of within-litter birth weight was indicated with a coefficient of variation for pup littermate birth weight. Coefficient of pup birth weight variation = standard deviation of litter birth weight/average litter birth weight. The pregnancy results are presented in Figure 1 and [Supplementary-material supplementary-material-1]. Within-litter birth weight variation was statistically lower in the GlcN supplement group than in the control group (5.55% for 0.5 mM GlcN, 5.77% for control group, respectively), and average litter weight of live-born rats in the 0.5 mM GlcN-supplemented group (2.27 ± 0.06) was significantly higher than that from the control group (2.02 ± 0.04). In addition, maternal placental efficiency (fetal body weight to placental weight ratio) was significantly increased in the 0.5 mM GlcN group (3.61 ± 0.11) in comparison with the control group (3.28 ± 0.08). The litter size of the 0.5 mM GlcN and the control group, respectively, was 13.45 and 11.73, while there was no significant difference.

RETRACTED

### 3.2. GlcN Supplementation before Mating Improved Ovary Weights of Rats

As shown in Table 1, both the absolute weight of ovary and relative weight of ovary in the GlcN supplementation group were higher than in the control group (*P* < 0.05) at the end of GlcN treatment (Table 1). Uterine weights were not statistically different between groups. There was no statistical difference in ADG, ADFI, and ADWI between the control and the GlcN groups ([Supplementary-material supplementary-material-1]).

### 3.3. GlcN Supplementation before Mating Improved Uniformity of Implantation of Rats

Embryonic implantation was investigated on the 6.5th day of pregnancy when blastocysts establish contact with the uterine endometrium. Rat dams fed GlcN had more implantation sites (15.75 ± 0.59, Figure 2(b)) compared with control dams (13.38 ± 0.63, Figure 2(a)). In the aspect of embryos distribution, extreme differences indicated as the number of implantation sites in two uterine horns were mainly observed in the control group. Expression levels of uterine receptivity-related genes were evaluated by quantitative real-time PCR. GlcN increased Alk3 (Figure 2(d)) and Bmp2 (Figure 2(e)) expressions in implantation sites and decreased IGF-1 (Figure 2(f)) and Mucin-1 (Figure 2(g)) levels. There was a tendency for iNOS expression to decline in the GlcN group.

### 3.4. GlcN Supplementation before Mating Changed the Maternal Hormones

The concentration of maternal reproductive hormones in plasma and biochemical parameters on D 19.5 is presented in Figure 3. In the GlcN group, progesterone, estradiol, and IGF-1 concentrations were significantly increased, while insulin (INS) and total cholesterol levels were decreased significantly in contrast with control dams. While there was no statistical difference in LDL-C, HDL-C, and triglyceride levels (Data are not shown).

## 4. Discussion

Currently, special attention has been given to great within-litter birth weight variation in litter-bearing animals, which is characterized by a higher proportion of low birth weight littermates [15, 16]. Low birth weight can result in poor postnatal survival and growth performance subsequently [16, 17]. Glucosamine has been increasingly reported to play important roles in oocyte maturation and early stages of embryo development [18]. Limited studies have focused on the impacts of GlcN supplementation before mating on embryo implantation and pregnancy. In the present study, we demonstrated, for the first time, that 0.5 mM GlcN administration before mating decreased the within-litter birth weight variation, while the average litter weight of live-born rats was increased, which is partly because of improved implantation as well as development of ovary through affecting maternal plasma hormones concentrations and uterine receptivity related gene expressions.

RETRACTED

As for the reproductive results, the within-litter birth weight variation was decreased, while the average litter weight was increased when 0.5 mM GlcN was supplemented before mating. Factors like ovulation rate, oocyte maturity, placental implantation ability, and placental transport efficiency could affect within-litter birth weight variation [15]. Glucosamine (GlcN) metabolism is closely related to oocyte maturation and early embryonic development through participating in the hexosamine biosynthesis pathway and activating the mTOR signal pathway [19]. GlcN is preferentially utilized as a substrate to form extracellular matrix hyaluronic acid, which is involved in the expansion of cumulus-oocyte complexes (COCs), mucification, and oocyte maturation *in vitro* [20–22]. The increased absolute and relative weight of the ovary indicated a better oocyte quality or more developed follicles in the GlcN group relative to controls [8]. Consistently, dams had a more efficient placenta (higher ratio of fetal body weight to placental weight) when administrated GlcN. Fetal development relies on the placenta to obtain nutrients and oxygen [23], especially during the rapid growth phase in the last third of gestation [24], and placental efficiency is related positively to reproductive performance [10]. In the present study, litter size did not markedly differ between the GlcN and the control groups. In contrast, several studies demonstrated an inhibitory effect of GlcN on litter size and embryo development. Tsai et al. [25] reported that litter size decreased when a sustained-release GlcN (15, 150 or 1500 *μ*g) was implanted into uterine horn ten days before coitus and during pregnancy compared with that in the placebo-implanted control group. Further, deteriorated implantation and reduced litter size on day 18 of gestation have been reported when 8-week-old mice were injected intraperitoneally with 20 or 400 mg/kg GlcN during periconception [26]. The difference between these observations and our results may be related to the much lower dose of GlcN used and different periods and route of administration.

RETRACTED

There were significant differences between maternal plasma metabolites in the GlcN group and the control group, which partly explained the reproductive results. Higher concentrations of progesterone and IGF-1 were detected in rats treated with GlcN compared with control dams. Progesterone is necessary for the maintenance of pregnancy. Consistently, total plasma cholesterol concentration in GlcN the group was reduced, which could result from enhanced utilization of cholesterol to synthesis steroid hormones. This explanation is supported by the fact that the levels of progesterone and estradiol were increased while LDL-C and HDL-C concentrations did not differ in dams treated with GlcN compared with controls. Glucosamine supplementation increased IGF-1 concentration which is important for embryonic development. IGF-1 is a major regulator of the growth rate and development of fetal [27–29].

Interaction between blastocysts and endometrium during the process of embryo implantation is a critical stage, which requires the involvement of both blastocyst and endometrial receptivity [8, 30]. Different blastocyst development ability may reduce the success rate of implantation. A large number of embryos were lost during the implantation period [31]. Based on better pregnancy results in GlcN supplemented group, we further evaluated the effects of GlcN on embryonic implantation. The results showed that the number of implantation sites increased with the improved uterine environment in the GlcN group, which indicated better blastocyst and endometrial receptivity.

We further assessed gene expression that is closely relevant to placental implantation. Bmp plays important roles in endometrium stromal cell decidualization via Alk3 signal, and Alk3 has been demonstrated necessary for the transition of the uterus from nonreceptive to receptive stages by inhibiting uterine epithelial cell proliferation during the window of implantation [32–34]. In this study, the expression levels of Alk3 and Bmp2 genes in implantation sites of the GlcN group were increased, and the levels of IGF-1 and Mucin-1 were decreased, which indicated that the uterine receptivity was improved. Decreased IGF-1 inhibits endometrium proliferation [35], and Mucin-1 is an E2-mediated gene. The downregulation of Muc-1 may be due to the attenuated response of endometrium to E2; it is consistent with what uterine environment needs to be switched from E2-dominant to P4-dominant stage. As indicated, the distribution of embryos in bilateral uterine horns in the control group was seriously unequal. A reasonable explanation for improved uterine receptivity is that blastocyst competence is more uniform in rats treated with GlcN [8].

RETRACTED

GlcN supplementation was conducted during the follicular phases of the estrous cycle, and its effects on within-litter variation and embryonic implantation seem to be closely related to the regulation of the ovaries development. Although several previous studies reported that the presence of glucosamine during maturation seriously interferes with the development of blastocysts *in vitro* [7], the relations between GlcN and oocyte maturation need further investigation *in vivo*.

## 5. Conclusions

Our study determined that GlcN supplementation before mating plays an important role in promoting the litter homogeneity, which is partly because of improved uterine receptivity. Our results provide a potential theoretical basis for formulating reasonable nutritional interventions to reduce the incidence of low birth weight animals, which will presumably improve the survival rate of newborns.

## Figures and Tables

**Figure 1:** Glucosamine (GlcN) supplementation before mating improves reproductive outcomes on day 19.5 of pregnancy. Fetal weight indicated body weight in late gestation (day 19.5 of pregnancy). Each icon in the figure represents the index of a litter of rats (*n* = 11 dams per group). (a) Within-litter birth weight uniformity, coefficient of pup birth weight variation (CV) = standard deviation of litter birth weight/average litter birth weight. (b) Average litter weight of live-born rats and (c) maternal placental efficiency were improved in the GlcN group compared with the control group. (d) Litter size (number of live-born rats) did not have a significant difference between groups. All data were represented as mean ± SEM. ^*∗*^There were statistically significant differences between groups when *P* value <0.05.

**Figure 2:** Effects of GlcN on implantation on day 6.5 of pregnancy. Distribution of implantation sites in the uterus in the control (a) and GlcN administration (b) groups. Implantation sites increased significantly in the GlcN groups compared with the control ones (c). The gene expression levels of Alk3 (d), Bmp2 (e), IGF-1 (f), Mucin-1 (g), and iNOS (h) in implantation sites were measured by quantitative real-time PCR. Data are expressed as mean ± SEM. ^*∗*^There were statistically significant differences between the two groups when *P* value <0.05.

**Figure 3:** GlcN alters maternal plasma progesterone (a), E2 (b), IGF-1 (c), insulin (d), and total cholesterol (e) concentrations on day 19.5 of pregnancy (*n* = 11). ^*∗*^There were statistically significant differences between the two groups when *P* value <0.05.

RETRACTED

**Table 1:** Organ index of rats at the end of GlcN treatment.

Items		Control	GlcN	*P* value
*Absolute organ weight (g)*				
Uterus		0.457 ± 0.073	0.431 ± 0.070	0.31
Ovary		0.145 ± 0.023	0.171 ± 0.026	0.01^*∗*^
*Relative organ index (%)*				
Uterus		0.208 ± 0.007	0.195 ± 0.003	0.16
Ovary		0.066 ± 0.003	0.079 ± 0.003	0.01^*∗*^

*n* = 10 dams per group. All data were presented as mean ± SEM. The relative organ index = organ weight/body weight *∗* 100%. ^*∗*^There were statistically significant differences between the two groups when *P* value <0.05.

## Data Availability

The data used to support the findings of this study are available from the corresponding author upon request.

## Supplementary Materials

Supplementary Materials The diet composition analysis is provided in Table S1. The concentration was determined on the basis of a gradient experiment which additionally included 1.0 mM GlcN and the results are presented in Table S2. A list of primer sequences is provided in Table S3. Growth performance during GlcN treatment periods is provided in Table S4.
